# Co-grafting of neural stem cells with olfactory en sheathing cells promotes neuronal restoration in traumatic brain injury with an anti-inflammatory mechanism

**DOI:** 10.1186/1742-2094-11-66

**Published:** 2014-04-02

**Authors:** Su-Juan Liu, Yu Zou, Visar Belegu, Long-Yun Lv, Na Lin, Ting-Yong Wang, John W McDonald, Xue Zhou, Qing-Jie Xia, Ting-Hua Wang

**Affiliations:** 1 Department of Histology, Embryology and Neurobiology, West China School of Preclinical and Forensic Medicine, Sichuan University, Chengdu, Sichuan 610041, China; 2 Institute of Neurological Disease, Translational Neuroscience Center, West China Hospital, Sichuan University, Chengdu, Sichuan 610041, China; 3 Department of Neurology, Johns Hopkins University School of Medicine, Baltimore, MD 21205, USA; 4 Institute of Neuroscience, Kunming Medical University, Kunming, Yunnan 650031, China

**Keywords:** Neural stem cells (NSCs), Olfactory en sheathing cells (OECs), Traumatic brain injury (TBI), Anti-inflammation

## Abstract

**Background:**

We sought to investigate the effects of co-grafting neural stem cells (NSCs) with olfactory ensheathing cells (OECs) on neurological behavior in rats subjected to traumatic brain injury (TBI) and explore underlying molecular mechanisms.

**Methods:**

TBI was established by percussion device made through a weight drop (50 g) from a 30 cm height. Cultured NSCs and OECs isolated from rats were labeled by Hoechst 33342 (blue) and chloromethyl-benzamidodialkyl carbocyanine (CM-Dil) (red), respectively. Then, NSCs and/or OECs, separately or combined, were transplanted into the area surrounding the injury site. Fourteen days after transplantation, neurological severity score (NSS) were recorded. The brain tissue was harvested and processed for immunocytochemistry, terminal deoxynucleotidyl transferase-mediated dUTP nick end labeling (TUNEL), and reverse transcription-polymerase chain reaction (RT-PCR).

**Results:**

Significant neurological function improvement was observed in the three transplant groups, compared to the TBI group, and co-transplantation gave rise to the best improvement. Morphological evaluation showed that the number of neurons in cortex from combination implantation was more than for other groups (*P* <0.05); conversely, the number of apoptotic cells showed a significant decrease by TUNEL staining. Transplanted NSCs and OECs could survive and migrate in the brain, and the number of neurons differentiating from NSCs in the co-transplantation group was significantly greater than in the NSCs group. At the molecular level, the expressions of IL-6 and BAD in the co-graft group were found to be down regulated significantly, when compared to either the NSC or OEC alone groups.

**Conclusion:**

The present study demonstrates for the first time the optimal effects of co-grafting NSCs and OECs as a new strategy for the treatment of TBI via an anti-inflammation mechanism.

## Background

Traumatic brain injury (TBI) occurs as a result of direct mechanical insult to the brain, and induces degeneration and death in the central nervous system (CNS) [1,2]. TBI is prevalent especially in male adolescents and adults, and severely affects the quality of peoples’ lives. Based on an epidemiological study in eastern China, traffic accidents, a blow or penetrating injury to the head, and falls from a high place were the primary causes of TBI, and their percentages were 60.9%, 13.4%, and 13.1%, respectively [3]. Among these, traffic accidents were the major cause for TBI in all age groups except for those over 75 years of age. For all patients, although 77.3% had good recovery, there was still a 10.8% mortality; 2.6% remained in a persistent vegetative state, 2.2% had severe disability, and 7.2% had moderate disability [4]. Much of this unfavorable outcome was due to secondary brain damage that occurred in the hours, days, and weeks after the primary insult [5]. Secondary cerebral injury was associated with impaired cerebral metabolism, hypoxia, and ischemia, which resulted in a complex, potentially irreversible pathophysiologic cascade of events. Currently, few interventions have been shown to be efficacious for the treatment of TBI in clinical trials [6], and it is therefore necessary to develop new therapeutic interventions for the clinical treatment of TBI.

Neural stem cells (NSCs) are characterized by their capacity for self-renewal and ability to differentiate into target cells [7]. It has been shown that transplanted NSCs can survive, differentiate into neurons and/or glia, and attenuate motor dysfunction after TBI [8,9]. These exciting advances in the stem cell field have boosted efforts to explore their therapeutic potential to ameliorate TBI deficits and efforts to elucidate their underlying molecular mechanism of action. However, the survival and differentiation of NSCs and their effect in traumatic brain is limited, and some new ways are needed to resolve these problems.

Olfactory en sheathing cells (OECs), as unique glial cells in the olfactory bulb and olfactory nerve, have properties of Schwann cells in promoting and assisting growth of axons [10-12]. Use of OECs in preclinical models of transplantation has been increasing in recent years. OECs not only promote long-distance regeneration of descending supraspinal and ascending propriospinal axons within both cord stumps of transected adult mammalian spinal cord [13], but can also successfully improve functional and structural recovery [14]. Importantly, OECs can act as bridges [15], and then release several cytokines that could promote neuronal survival and neurite outgrowth following injury. Therefore, OECs transplants might be considered as a supporting strategy for NSCs survival and for enhancing NSCs effects for lasting functional recovery in a traumatic milieu in the adult mammalian CNS.

In the present study, we aimed to investigate functional improvement and associated anti-inflammatory mechanisms involving the cytokines IL-1 and IL-6 following a combination graft of NSCs and OECs in TBI rats. The study could suggest new strategies for co-grafting of NSCs and OECs to promote functional recovery of TBI rats, and could elucidate underlying mechanisms. The results could be useful for the treatment of patients with TBI in future clinical trials.

## Methods

### Cell culture, characterization, and transplantation

NSCs were obtained from hippocampus of rat embryos [16]. They were cultured in a standard medium containing a mixture of Dulbecco’s modified Eagle’s medium (DMEM) and Ham’s F-12 medium, supplemented with 1% N_2_, 20 μg/L basic fibroblast growth factor (bFGF), 2 mmol/L glutamine, 10,000 U/L penicillin, and 10 mg/L streptomycin. The cultures were kept in a standard humidified air incubator containing 5% CO_2_ and maintained at 37°C. They were divided when the cells reached approximately 90% confluence. After passage, a portion of the single cell suspension was plated onto poly-L-lysine-coated glass cover slips or plastic culture dishes at a density of 10^5^ cells/mL of medium. Twelve hours after plating, a portion of the cells was fixed in 4% paraformaldehyde for 20 min and washed with PBS three times. For immunocytochemistry, cover slips were washed in PBS and incubated in 1% H_2_O_2_ in PBS for 20 min. The cells were permeabilized and pre-incubated with blocking solution (containing 2% goat serum, 0.3% Triton X-100, and 0.1% BSA in PBS) for 30 min at room temperature. They were then incubated overnight with a primary antibody (nestin, 1:200, Millipore Bioscience Research Reagents, Temecula, CA, USA) diluted in the same blocking solution at 4°C, washed with PBS, and incubated with secondary antibodies diluted in the same blocking solutions for 30 min at 37°C. Then, the cells were observed with a light microscope (Leica, Solms, Germany). OECs were obtained from neonatal rat olfactory bulb and purified as described before [12]. After purification, a portion of the cultured OECs were fixed and processed for immunocytochemistry to detect the specific antigen rat anti-p75-NGFR (low-affinity nerve growth factor receptor, p75, 1:400, Abcam, Cambridge, UK), using a two-step method described previously [12].

### Animals, surgical procedures, and transplantation

All protocols involving the use of animals were in compliance with the National Institutes of Health Guide for the Care and Use of Laboratory Animals, and were approved by the Animal Care and Use Committee, Sichuan University, Chengdu, China. Female Sprague-Dawley (SD) rats weighing about 200 ± 20 g were used in the study (Table 1). They were randomly assigned to five groups: a sham-operated group (rats with skull exposed but not subjected to weight impaction, and receiving saline injections instead of cultured cells); a TBI group (rats subjected to TBI and receiving saline treatment); an NSC group (rats subjected to TBI and receiving NSCs transplantation); an OEC group (rats subjected to TBI and receiving OECs transplantation); and a co-transplantation group (rats subjected to TBI and receiving co-transplantation of both NSCs and OECs).

**Table 1:** Animal numbers in each procedure

**Group**	**Behavior test (7 and 14 days)**	**Apoptosis assessment (7 days)**	**Gene expression detection (7 days)**
Sham	6	3	6
TBI	6	3	6
NSC	7	3	6
OEC	8	3	6
NSC + OEC	6	3	6

*NSC*, neural stem cell; *OEC*, olfactory en sheathing cell; *TBI*, traumatic brain injury.

For the TBI model, rats were anesthetized by intraperitoneal injection of 3.6% chloral hydrate (1 mL/100 g). The scalp was incised on the midline, exposing the skull. A 5 mm hole was drilled into the right parietal bone, not touching the dura mater. A 50 g-weight hammer was allowed to fall from a 30 cm height along guide stick to create a contusion brain injury model. At the end of the procedure, the exposed dura was covered with bone wax and the scalp sutured. The rats were placed in a warmed, oxygenated recovery chamber with free access to food and water under controlled temperature (24 ± 21°C) and humidity (55 ± 5%) as well as a 12/12 h light–dark cycle. Postoperative care included injections of penicillin to prevent infection.

Before transplantation, the cells from a third passage were trypsinized (0.125% trypsin, 5 min), and gently titrated into serum containing medium to inactivate the trypsin, then washed three times by gently pelleting the cells, followed by a low-speed centrifugation (900 *g*). They were resuspended in DMEM/F-12 to yield/reach a final concentration of 1 × 10^7^ cells/mL. Trypan blue was used to assess their viability. The suspension was kept on ice and gently triturated before each injection to keep the suspension dispersed and free of cell clumps. NSCs and OECs were labeled with Hoechst 33342 and CM-Dil, and then engrafted into tissues around the injury site through the microinjection needle of a stereotaxic instrument. Four injections were made, each containing 5.0 μL of suspended cells, delivered at 1 μL/min. For the co-grafting group, 50% NSCs and 50% OECs were injected, suggesting that the total number of cells for each treatment was the same. Sham-operated animals and TBI control animals received only saline injections.

All transplant recipients received 10 mL of cyclosporine each, administered intraperitoneally, beginning 3 days before transplantation and continuing for 1 week.

### Assessment of neurological function

Neurological function was evaluated by a modified neurological severity score (NSS) on the day before, and on days 7 and 14 after transplantation [17]. The evaluations consisted of motor (muscle status, abnormal movement), sensory (visual, tactile, proprioceptive), reflex, and balance tests; and were recorded on a scale of 0 to 18 (normal score, 0; maximal deficit score, 18). They were performed by blinded, trained observers. For the NSS, 1 point was scored for inability to perform the test or the lack of a tested reflex. Thus, a higher score would point to a more severe injury. All rats were given enough time to become familiar with the testing environment before inflicting the brain injury. This was assessed by the rat’s ability to perform all the tests, and then an NSS was assigned.

### Tissue preparation

For assessment of terminal deoxynucleotidyl transferase-mediated dUTP nick end labeling (TUNEL) staining and reverse transcription-polymerase chain reaction (RT-PCR) 1 week after TBI, and for behavior immunohistochemistry 2 weeks after TBI, rats were anaesthetized and tissues further processed. For TUNEL and immunostaining, a total of 500 mL of 0.1 M/L PBS (pH 7.2 to 7.3, room temperature) was introduced into the left ventricle for 20 to 30 min, followed by 500 mL of 4% paraformaldehyde in 0.1 M/L PBS (pH 7.2 to 7.3, 4°C for 1 h). The brain was removed and immersed in the same fixative for 4°C for 24 hours, and then transferred to PBS containing 30% sucrose before cryosectioning. Serial sections of the brain tissues were sliced at a thickness of 30 μm using a cryotome (CM1900, Leica), and mounted on gelatin-pretreated slides. For RT-PCR, the brain tissues were directly harvested without perfusion, then frozen and kept at -80°C until used.

### Survival and differentiation of grafted cells

Grafted cell survival was assessed by identifying fluorescent cells under fluorescence microscopy in brain sections. Three microscopic fields (400×) from each section of each rat in each group were acquired to perform subsequent statistical analysis. Differentiation of NSC-derived cells in the host brain was detected by fluorescence immunohistochemistry staining. The antibodies used included NeuN (for neuronal differentiation), GFAP (for astrocyte differentiation), and APC (for oligodendrocyte differentiation), respectively. In the above procedures, mouse anti-NeuN (1:1,000, Millipore Bioscience Research Reagents), rabbit anti-GFAP (1:200, Millipore Bioscience Research Reagents), and mouse anti-APC (1:200, Millipore Bioscience Research Reagents) were used, followed by routine immunoenzyme-linked immunocytochemistry.

### Neuronal survival

To detect neuronal survival in brain, sections from tissue surrounding the injured brain were evaluated using routine immunofluorescence staining. The primary antibody was NeuN (1:1,000, Millipore Bioscience Research Reagents) and the second antibody was conjugated with Cy3 (red) fluorescent. For control, the primary antibody was omitted for all markers. Labeled cells and regenerating axons were examined with a fluorescence microscope.

### TUNEL staining

TUNEL was used to detect apoptotic neurons in the host brain. For each rat, the brain tissues sectioned at 20 μm thickness were stained with TUNEL reagents according to the manufacturer’s instructions. The sections were dried, rehydrated in PBS, and treated with proteinase K for 5 min at room temperature. After quenching the endogenous peroxidase activity with 3% H_2_O_2_ in methanol, the sections were successively treated with an equilibration buffer, working TdT enzyme for 4 h at 37°C and blocking buffer. Finally, the reaction was visualized by streptavidin-biotin-peroxidase complex and diaminobenzidine. Sections incubated without the enzyme were used as negative controls. There were two distinct patterns of TUNEL staining, as reported previously [18]. Some cells were densely labeled and showed clear apoptotic characteristics, such as perinuclear ring formation, patches, or an apoptotic body. Other cells were weakly labeled and considered to be necrotic cells. Only the densely labeled cells were counted as TUNEL-positive cells [19]. In order to compare the numbers of apoptotic cells, three fields (400×) from each section of each rat in each group were taken for statistical analysis.

### RT-PCR

To explore the molecular mechanism underlying the restorative features observed in the host brain following transplantation, the expressions of IL-1, IL-6 (inflammatory factors), and BAD (apoptosis signal molecule) were determined. Total RNA from pericontusional tissues of each group was extracted using a commercially available kit (Fermentas, Burlington, ON, Canada). The procedure followed the manufacturer’s instructions. In order to remove any contaminating genomic DNA, samples were incubated at 37°C for 40 min with DNase I, followed by DNase inactivation with a DNase inactivation reagent. For reverse transcription, 2.0 μg RNA per sample was reverse transcribed using a reverse transcription kit in a total volume of 50 μL according to the manufacturer’s instructions. cDNA was diluted in TE buffer, aliquoted, and stored at -20°C. Primers for IL-6, BAD, and β-actin (as an internal control) were designed with the primer 5.0 software and then empirically tested. IL-1β (234 bp), forward GAGCTGAAAGCTCTCCACCT and reverse TTCCATCTTCTTCTTTGGGT; IL-6 (378 bp), forward CTTGGGACTGATGTTGTTGA and reverse CTGGCTTTGTCTTTCTTGTTAT; and BAD (435 bp), forward CGAGTGAGCAGGAAGACGC and reverse AATTTCGATCCCACCAGGAC. β-actin (227 bp), forward GTAAAGACCTCTATGCCAACA and reverse GGACTCATCGTACTCCTGCT. PCR semi-quantitative conditions were optimized by varying the amount of template and cycle number to determine a linear amplification range. Following PCR, the product was electrophoresed on a 1.5% agarose gel, post-stained with gold view, and identified by size. The optical density (OD) of each product band, including the objective gene and β-actin was obtained, and the OD ratio between investigated genes and β-actin were calculated to semi-quantify the objective gene level.

### Statistical analysis

Statistical analysis was conducted using SPSS 16.0 software (SPSS Inc., Chicago, IL, USA). The measurement data are expressed as mean ± SD and were subjected to statistical analysis using one-way analysis of variance (ANOVA). When significant interactions were detected in any ANOVA paradigm, post-hoc Student-Newman-Keuls *t*-tests were used to demonstrate effects between individual groups. Values of *P <*0.05 were considered statistically significant.

## Results

### Characterization of cultured cells

After 2 to 3 days of culture, cultured cells began to form neurospheres and showed increases in number and size by 5 days (Figure 1A). The cells stained with nestin were confirmed as NSCs (Figure 1B). These cells emitted blue fluorescence after Hoechst 33342 labeling under fluorescence microscopy (Figure 1C). OECs were successfully isolated and assumed a shuttle appearance (Figure 1D), and were identified by p75 immunostaining (Figure 1E) confirming that they were OECs. In order to track the transplanted OECs, CM-Dil was used to label OECs, as shown in Figure 1F.

**Figure 1:** ***In vitro *characterization of NSCs and OECs.** Representative images of NSCs and OECs *in vitro*. **(A)** NSCs are tighter and larger 5 days after isolation from rat hippocampus, **(B)** nestin + neurosphere formation, and **(C)** neurons labeled with Hoechst 33342. **(D)** OECs present bipolar and multipolar cells with a three-dimensional, interlaced network after purified culture, **(E)** NGFR-p75+, and **(F)** labeled with CM-Dil. Scale bars are 30 μm in **(A)** and 50 μm in **(D)**. CM-Dil, chloromethyl-benzamidodialkyl carbocyanine; NSC, neural stem cell; OEC, olfactory en sheathing cell.

### Character of differentiation of NSCs

Immunocytochemistry staining was used to detect differentiation of NSCs into neurons (NeuN-positive), oligodendrocytes (APC-positive), and astrocytes (GFAP-positive) (Figure 2A, B, C, D). *In vitro*, NSCs exhibited the capacity to differentiate into neurons, astrocytes, and oligodendrocytes. NSC, neural stem cell.

**Figure 2:** ***In vitro *characterization of NSC differentiation.** NSCs isolated from rats differentiate into neuron-like cells and glial cells, and express **(A)** NeuN (a neuron marker), **(B)** GFAP (an astrocyte marker), and **(C)** APC (an oligodendrocyte marker) as shown by immunocytochemical staining. **(D)** Quantitative differentiation (percent of NSCs). Scale bar = 100 μm, shown in **(C)**. NSC, neural stem cell.

### NSS

Before TBI or sham operation, rats received a score of 0 and showed normal cerebral function. However, after TBI surgery, the rats showed impairment of locomotor functions and the NSS significantly increased when compared to the sham group (*P* <0.01). In addition, separate or combined transplantation of NSCs and OECs resulted in prominent decreases in the NSS, suggesting a significant improvement of neurological function (*P* <0.05; Figure 3).

**Figure 3:** **Functional assessment for behavior after cell transplantation.** NSS tests 7 and 14 days after TBI surgery show that the scores significantly increased immediately after TBI (*P* <0.01 versus sham). However, compared with the TBI group 7 and 14 days after the injury, the NSS of rats that received separate or combined transplantation of NSCs and OECs significantly decreased (*P* <0.05), and the scores in co-grafted rats are even lower (*P* <0.05). *Statistical significance of *P* <0.05. ^#^Statistical significance of *P* <0.01. NSC, neural stem cell; NSS, neurological severity score; OEC, olfactory en sheathing cell; TBI, traumatic brain injury.

### Survival and integration of grafted cells in host tissues

Cells emitting blue fluorescence were found in pericontusional tissue, confirming these as transplanted NSCs (Figure 4A, B), while those emitting red fluorescence were identified as OECs (Figure 4C, D). This confirmed that grafted cells could survive and migrate around the injury site. Given that only half the number of NSCs were transplanted in the co-grafting group compared to the NSC group at the beginning of cell transplantation, it is clear that the number of surviving NSCs after co-grafting is 3.4-fold (68/20) higher compared with NSCs only transplantation into the brain. Moreover, compared with NSCs implanted alone, the number of surviving NSCs in the co-transplantation group is significantly increased (*P* <0.05; Figure 4E). This finding demonstrates that OECs play an important role in enhancing the survival of NSCs.

**Figure 4:** ***In vivo *survival and integration of transplanted cells. (A, B)** Transplanted cells emit blue fluorescence and are observed in the pericontusional brain tissue of rats, which suggests grafted NSCs can survive in host tissue. **(C, D)** Similarly, transplanted CM-Dil-labeled OECs survive in the brain tissue of rats. **(E)** Combined transplantation of NSCs and OECs increases the number of surviving NSCs (*P* <0.05 versus NSC group). Scale bars = 100 μm, shown in **(A)** and **(C)**. *Statistical significance of *P* <0.05. CM-Dil, chloromethyl-benzamidodialkyl carbocyanine; NSC, neural stem cell; OEC, olfactory en sheathing cell.

### Neuronal survival in host brain

In the sham-operated group, neurons presented a healthy and robust appearance (Figure 5A). After TBI, neurons surrounding the lesion site appeared shrunken and were significantly reduced in number when compared with the sham-operated group (Figure 5B). Notably, NSCs or OECs grafting brought about a significant increase in the number of neurons (Figure 5C, D). Co-grafting of NSCs and OECs resulted in the largest number of surviving neurons (*P* <0.05 versus NSC group; *P* <0.05 versus OEC group; Figure 5E).

**Figure 5:** **Neuronal survival in host brain. (A, B, F)** The number of neurons labeled by NeuN in host brain significantly decreases following TBI when compared with sham (*P* <0.05). **(B, C, D, E, F)** However, separate or combined transplantation of NSCs and OECs increases neuronal number (*P* <0.05 versus TBI). **(C, D, E, F)** Furthermore, co-grafting group resulted in the highest number of surviving neurons; higher than the NSC only group or the OEC only group (*P* <0.05). Scale bars = 100 μm, shown in **(A)**. *Statistical significance of *P* <0.05. NSC, neural stem cell; OEC, olfactory en sheathing cell; TBI, traumatic brain injury.

### Neuronal apoptosis

TUNEL staining showed the presence of apoptotic cells with typical dark brown, rounded, or oval apoptotic bodies. Compared with the sham-operated group (Figure 6A), the number of apoptotic neurons in the brain significantly increased following TBI surgery (*P* <0.01). However, separate or combined transplantation treatment resulted in a significant decrease in the number of apoptotic cells (*P* <0.05 versus TBI; *P* <0.01 versus TBI; Figure 6B, C, D, E, F). Moreover, compared with separate transplantation of NSCs or OECs, the number of apoptotic cells decreased significantly in the co-grafted group (*P* <0.05; Figure 6C, D, E, F).

**Figure 6:** **Neuronal apoptosis in host brain. (A, B, F)** TUNEL staining shows that neuronal apoptosis increased significantly after TBI (*P* <0.01 versus sham group), **(B, C, D, E, F)** whereas separate or combined transplantation of NSCs and OECs has a reverse effect on neuronal apoptosis (*P* <0.05 versus TBI; *P* <0.01 versus TBI), and **(C, D, E, F)** results with co-grafting are the best (*P* <0.05 versus NSC; *P* <0.05 versus OEC). Bars = 100 μm, shown in **(A)**. *Statistical significance of *P* <0.05. ^#^Statistical significance of *P* <0.01. NSC, neural stem cell; OEC, olfactory en sheathing cell; TBI, traumatic brain injury; TUNEL, terminal deoxynucleotidyl transferase-mediated dUTP nick end labeling.

### RT-PCR

To address the molecular mechanism for cell transplantation, the expressions of IL-1β, IL-6, and BAD genes were detected in the brain of rats subjected to TBI. Of note, although there is no statistical difference in expression of IL-1β following the different administrations, mRNA expression of IL-6 and BAD in the co-transplantation group exhibited a significant down-regulation in pericontusional regions at 7 days when compared with the OEC group (*P* <0.05; Figure 7A, B). Similarly, BAD gene expression was significantly reduced in the NSC + OEC group compared with the TBI group or the NSC only group, (*P* <0.05; Figure 7A, B). This suggests that co-graft effects on behavior and anti-apoptosis may be linked to down-regulation of IL-6 and BAD.

**Figure 7:** **Changes of gene expression after cell transplantation.** Gene expression of IL-1β, IL-6, and BAD in host brain were examined by **(A)** RT-PCR and **(B)** quantitative analysis. Although IL-1β gene expression is not statistically different after cell transplantation, IL-6 gene expression significantly decreased in the pericontusional regions of the co-transplantation group at 7 days compared with OEC only grafts (*P* <0.05). Moreover, BAD gene expression decreased significantly in the NSC + OEC group when compared with that of the TBI, NSC, and OEC groups (*P* <0.05). *Statistical significance of *P* <0.05. NSC, neural stem cell; OEC, olfactory en sheathing cell; TBI, traumatic brain injury.

## Discussion

This study demonstrates that intracerebral implantation of NSCs and OECs after TBI effectively enhances survival of NSCs and improves neurological function. Moreover, co-grafting had the best results in attenuating posttraumatic neuronal apoptosis, compared with the single NSCs or OECs grafting. This could be associated with the observed down-regulation of IL-6 and BAD genes in the posttraumatic period.

### Effects of grafts on behavior and morphology

NSCs transplanted into host tissue can produce neuroactive substances [20], which are important for neuronal survival and axonal growth [21,22]. However, in the injured milieu, survival of NSCs encounters challenges. As a result, additional supportive strategies to maintain NSCs survival are necessary. OECs, as a unique type of glial cell that arises from the neural crest, exhibit the ability to secrete several growth factors, and could therefore serve as support cells for NSCs survival. In our study, engrafted OECs survived and migrated together with NSCs in brain. They therefore may provide a favorable cellular substrate with molecules that could facilitate axonal binding and extension and neurotropic effects [23] for neuronal survival. In addition, OECs may be useful in myelin development or remyelination [24,25], and even in promoting axonal growth [21,23]. In this study, engrafted NSCs and OECs were well integrated into the host and enhanced structural and functional restoration in rats following TBI. Co-transplantation may be considered as a new strategy for the treatment of TBI.

### Possible mechanism for structural restoration following co-grafting

The exact mechanism by which co-transplantation brings about functional restoration after TBI is unclear. An increase in neuronal survival may play an important role in this process. Other important events may include angiogenesis, formation of new synaptic junctions, and structural reorganization, as reported previously [15]. In our study, co-transplantation of NSCs and OECs exerted synergistic effects in amelioration of TBI, which may involve the following: 1) addition of OECs enhanced survival of NSCs, which is beneficial to structural restoration; 2) NSCs and OECs could secrete many types of growth factors that are useful for the formation of new synaptic junctions, and anti-apoptosis; 3) after TBI, lost neurons might be replaced by engrafted NSCs, while OECs could serve as ‘bridges’ to guide axonal elongation, or could promote myelination [24]; and 4) co-grafting may down regulate expression of cytokines, such as IL-6, and decrease BAD levels, so as to protect neurons from apoptosis via an anti-inflammatory mechanism.

### Implications of down-regulation of IL-6 and BAD genes

In the investigation of mechanisms of cell death and survival, apoptosis genes and neurotrophic factors are commonly considered. However, the present study mainly shows that co-transplantation of NSCs and OECs can regulate expression of IL-6, in addition to BAD, a crucial molecular signal involved in anti-inflammatory effects and apoptosis. IL-6 was originally identified as a major inducer of immune and inflammatory responses under injury conditions [26]. IL-6 *in vitro* enhances glutamate-mediated excitotoxicity in cerebellar granule cells, and can cause blood–brain barrier damage *in vivo*[27]. Transgenic mice overexpressing IL-6 display gliosis, neuronal cell loss, and learning disabilities with prominent neurodegeneration [28]. Hence, excessive IL-6-mediated inflammation is likely to play a fundamental role in the pathogenesis of the undesirable outcomes of TBI. In this study, we found that co-grafts could down regulate expressions of the inflammatory cytokine IL-6 but not IL-1β. This suggests that IL-6 may be a vital molecule in TBI following co-grafting. In addition, BAD, as a pro-apoptotic protein in the mitochondria-mediated apoptosis pathway [29,30], was also involved. The apoptotic activity of BAD is dependent on its phosphorylation status at Ser112, Ser136, and Ser155 [31]. When BAD is phosphorylated at these sites, it forms a complex with 14-3-3 proteins that cannot induce apoptosis [32]. In our study, BAD expression was greatly down regulated following co-transplantation. This could certainly lead to reduced apoptotic activity. Hence the prevention of cell apoptosis by the co-graft could be dependent on BAD regulation, a vital apoptosis signal molecule.

## Conclusions

The present study provides new evidence to confirm the effects of co-grafting of NSCs and OECs in TBI rats, as demonstrated by restored structural integrity, attenuated neuronal apoptosis, promotion of host neuronal survival, and down-regulation of the expression of IL-6 and BAD genes in TBI rats. These findings could be useful in suggesting new strategies for treatment of TBI, and provide insight into potential underlying mechanisms.

## Abbreviations

ANOVA: Analysis of variance; bFGF: Basic fibroblast growth factor; BSA: Bovine serum albumin; CM-Dil: Chloromethyl-benzamidodialkyl carbocyanine; CNS: Central nervous system; DMEM: Dulbecco’s modified Eagle’s medium; IL: Interleukin; NSC: Neural stem cell; NSS: Neurological severity score; OD: Optical density; OEC: Olfactory en sheathing cell; PBS: Phosphate-buffered saline; RT-PCR: Reverse transcription-polymerase chain reaction; SD: Sprague-Dawley; TBI: Traumatic brain injury; TUNEL: Terminal deoxynucleotidyl transferase-mediated dUTP nick end labeling.

## Competing interests

The authors declare that they have no competing interests.

## Authors’ contributions

THW, QJX, and SJL designed the study. SJL, YZ, QJX, LYL, XZ, NL, and TYW performed the experiments. SJL, VB, and JM discussed the results and prepared the manuscript. All authors read and approved the final version of the manuscript.
